# The Current Antimicrobial and Antibiofilm Activities of Synthetic/Herbal/Biomaterials in Dental Application

**DOI:** 10.1155/2022/8856025

**Published:** 2022-08-02

**Authors:** Ali Moghaddam, Reza Ranjbar, Mohsen Yazdanian, Elahe Tahmasebi, Mostafa Alam, Kamyar Abbasi, Zahra Sadat Hosseini, Hamid Tebyaniyan

**Affiliations:** ^1^Research Center for Prevention of Oral and Dental Diseases, Baqiyatallah University of Medical Sciences, Tehran, Iran; ^2^School of Dentistry, Baqiyatallah University of Medical Sciences, Tehran, Iran; ^3^Department of Oral and Maxillofacial Surgery, School of Dentistry, Shahid Beheshti University of Medical Sciences, Tehran, Iran; ^4^Department of Prosthodontics, School of Dentistry, Shahid Beheshti University of Medical Sciences, Tehran, Iran; ^5^Department of Genetics and Biotechnology, School of Biological Science, Varamin-Pishva Branch, Islamic Azad University, Tehran, Iran; ^6^Science and Research Branch, Islamic Azad University, Tehran, Iran

## Abstract

Herbal and chemical products are used for oral care and biofilm treatment and also have been reported to be controversial in the massive trials conducted in this regard. The present review is aimed at evaluating the potential of relevant herbal and chemical products and comparing their outcomes to conventional oral care products and summarizing the current state of evidence of the antibiofilm properties of different products by evaluating studies from the past eleven years. Chlorhexidine gluconate (CHX), essential oils (EOs), and acetylpyridinium chloride were, respectively, the most commonly studied agents in the included studies. As confirmed by all systematic reviews, CHX and EO significantly control the plaque formation and gingival indices. Fluoride is another interesting reagent in oral care products that has shown promising results of oral health improvement, but the evidence quality needs to be refined. The synergy between natural plants and chemical products should be targeted in the future to accede to the formation of new, efficient, and healthy anticaries strategies. Moreover, to discover their biofilm-interfering or biofilm-inhibiting activities, effective clinical trials are needed. In this review article, therapeutic applications of herbal/chemical materials in oral biofilm infections are discussed in recent years (2010-2022).

## 1. Introduction

Skin, respiratory and gastrointestinal mucosa, and the oral cavity which covers most of the surface of the human body are colonized by bacteria and provide a specific environment for microorganisms [1]. Oral biofilm or dental plaque in the oral cavity of all mammals is one of the prime examples that is detected to be hosting seven hundred specific bacterial species [2]. As a dynamic microbial biofilm, dental plaque consists extracellular matrices (ECM) and numerous bacterial species containing common and pathogenic microorganisms [1]. In addition to bacteria, the oral cavity of the human contains hundreds of various viral and fungi species. Generally, there may be over 10^11^ microorganisms per milligram of dental plaque which can cause different dental pathologies including gingivitis, caries, and periodontitis. Biofilm-originated infections can lead to fundamental issues in society in terms of economical and health aspects [3]. Biofilms usually consume natural teeth and dental prosthesis materials including either dentures or implants, as well as organic acids as the substrates. The increased secretion of organic acids is attributed to the consumption of carbohydrate-rich food. With increasing oral bacterial colonization, the extracellular polymeric substance (EPS) such as polysaccharide alginate is also overproduced [2]. Such substance provides a mucoid biofilm that facilitates developing resistance to antibiotics and the host's immune response [4]. As a result, the risk of chronic infections raises and their treatment becomes more difficult. Untreated infection for any reason causes enamel demineralization and dental caries [2, 4]. Dental caries and periodontal problems are common mouth and tooth diseases all over the world that affect almost every age and geographic communities [2]. In Europe, the incidence of dental caries is about 20-90 % in children at 6 years old and very close to 100% in adults. In the same population, 0.5-3.5 teeth of children at age 12 are conflicted by dental caries on average. Besides, the rate of severe periodontal (gum) disease in adults at middle ages and more advanced ages is 5-20% and 40%, respectively. In addition, people about 30% of the population have no natural teeth [5]. The loss of natural teeth due to dental caries and severe periodontal diseases can substantially affect the patients' tooth function and reduce their quality of life [5]. As a preventive strategy, the biofilms should be controlled appropriately to inhibit their physiological heterogeneity and interactions from developing dental mineralization and systemic inflammation [6]. The relationship between prosthetic loading or bacterial infection and implant failure has been indicated in the literature. The prevalence of mucositis and peri-implantitis has been reported to be around 30% and 9%, respectively [7]. This high prevalence of oral biofilm-related infectious diseases necessitates developing new and more effective treatments; as such in the US, over $81 billion are spent annually on such research [8]. The accessibility and highly multibacterial environment of the mouth make it a suitable setting for studying new modalities of biofilm inhibition. Results from studies on the oral cavity can be also extended to other biofilm-associated issues pertaining human health or industrial purposes [8]. Despite the difficulties of biofilm eradication, through decades, several conventional strategies have been applied to control dental biofilms. A popular example is brushing as a mechanical method that can effectively remove biofilms. This physical method is a common and important way to remove biofilms from dentures and prevent infection but not enough. Evidence shows that for controlling the oral biofilms, some form of chemical and biological cleanser is also required [9]. Alkaline peroxides, in the form of tablets, are a common popular approach to clean dentures. When these tablets are added to water, an effervescent alkaline solution is produced that generates hydrogen peroxide and active oxygen that penetrate to areas not accessible for brush and clean them [10]. Antiplaque oral rinses play an important role in biofilms. Although rinses containing chlorhexidine gluconate and essential oils can effectively remove plaques, they may have unwanted side effects too. However, such chemicals can be associated with side effects such as tooth discoloration and occasional loss of taste. Therefore, essential oils are increasingly being conveyed and preferred as alternatives with low mammalian toxicities and side effects [11]. Because of the side effects and limited efficiency of classic chemicals in oral planktonic and biofilm eradication, the search for novel nature-inspired antibiofilm methodologies continues. In this regard, the note of Hippocrates saying “nature itself is the best physician” has been updated to the importance of the plant kingdom against biofilm-related dental diseases [12–14]. Then, in addition to using some enzymes for degrading the protein matrices of biofilm, several naturals, herbal-based materials, or natural plant extracts have been added to some mouth rinse formulations for their anti-inflammatory and antimicrobial properties [11, 15]. Some herbal species with antiplaque properties existing in commercially available products are *Centella asiatica*, *Echinacea purpurea*, and *Sambucus nigra* [15]. Another example is naturally derived polyphenols that are being extensively discussed in scientific studies for their preventive and/or treating effects on many chronic infection/inflammatory-based diseases such as cardiovascular, metabolic, or neurodegenerative disorders and cancers, as well as oral diseases [16]. It is hoped that some of the materials discussed in this article will be able to be employed in dental research and industry, such as the development of dental sealers, lingual cements (are used in clinical dentistry to seal), biocompatible, bacteriostatic, nonshrinking, and nondispersible sealers are ideal for use, so that if a sealer was to extrude from the canal, it could be dissolved without causing damage to the tissue. Regardless of the type of root canal sealer used, all root canal sealers contain a certain level of toxicity. Therefore, even though newer sealers have been introduced that have been deemed highly biocompatible as a result, there is still a concern about their cytotoxicity. There have been numerous studies examining dental materials' cytotoxicity, especially soft tissues [17, 18]. In this review article, therapeutic applications of herbal and chemical materials in oral biofilm therapy in *in vitro*, *in vivo*, and clinical studies are discussed in the recent decade (2010-2022).

## 2. Research Methodology

In this review article, a comprehensive overview of the most important and critical aspects of the topic's knowledge is discussed. Several synthetic/herbal/biomaterials were investigated for their antimicrobial and antibiofilm activities. A search was performed on PubMed (2010–2022) using the keywords: (oral biofilm) OR (dental biofilm) AND (herbal treatment) AND (chemical treatment). A variety of sample types, microorganism species, methods, types of studies (in vitro, in vivo, and clinical), and results were evaluated in the studies.

## 3. Biofilm

### 3.1. Biofilm and Diseases

Similar to growth regulation, heterogeneity, proteolytic systems, and encapsulation in a self-created polymeric matrix, plaque formation is a survival mechanism taken by pathogenic microbes for adapting to stress conditions and host immunological responses. Biofilm formation is affected by the colonization area and matrix. Besides an important physical barrier against drugs, matrix provides a protective ecological niche for single or consortia microorganisms of several species to survive and/or cause diseases. The pathogenic species developing biofilms usually include fungal species (e.g., *Candida albicans*), gram-positive bacteria (e.g., *Staphylococcus epidermidis, Mycobacterium tuberculosis*, and *Mycobacterium abscessus*), and gram-negative bacteria (e.g., *Pseudomonas aeruginosa*) as well as *Mycoplasma pneumonia* that can develop resistance against immune responses and drug leading to serious health concerns [19]. Regarding the endodontic, *Enterococcus faecalis* (*E. faecalis*) is the leading pathogenic agent specifically in secondary and persistent infections [20].

### 3.2. Biofilm Formation

Microbes can form biofilms on almost any surface generally through a sequence of attachment and assembling micro colonies that leads to a differentiated mature structure. Attachment involves bacterial deposition and adhesion by anchoring either of matrix or earlier colonies. Sedimentation, hydrodynamic forces, and Brownian motion account for deposition while intermolecular forces such as acid-base, Lifshitz–Van der Waals, hydrophobic, and electrostatic interactions manage bacterial adhesion to the substratum. OmpA, fibronectin-binding proteins (FnBPs), protein A32, SasG, and biofilm-associated protein (BAP) are other surface-associated proteins that contribute to the microorganismal attachment as the initial stage of biofilm formation [21]. Another main mechanism underlying biofilm formation is quorum sensing (QS) which is a cell-to-cell communication mechanism and has been detected almost in all microorganismal species including gram categories (Figures 1 and 2). Quorum sensing involves small signaling molecules that mediate colonization and control biofilm formation whose disassembly or dispersion only takes place through mechanical and active processes [21]. Resistance to bactericidal or bacteriostatic agents commonly occurs in planktonic cultures at concentrations normally inhibitory [22]. Describe resistance as the mechanisms through which an antimicrobial agent is prevented from interacting with its intended target [23]. Mutations and transfections (interspecies exchange of antibiotic resistance genetic elements) are the main mechanisms recognized as responsible for acquired resistance; however, some species have intrinsic resistance and phenotypes based on their wild-type genes. For example, gram-negative bacteria are intrinsically more resistant to antibiotics because of their less impermeable outer membrane. Accordingly, some biofilm-based resistance mechanisms such as antibiotic efflux pumps, matrix *β*-lactamases, and antibiotic sequestering molecules (such as eDNA and NdvB-derived periplasmic glucans) are discussed in this review [23].

### 3.3. Oral Biofilm

In the past 100 years, medical literature contained considerable interest toward bacteria at their planktonic phase presenting in host's mouth, while today, we know that oral microbiota is generally organized as biofilms [24]. The humidity, temperature, and nutrient-rich environment of the oral cavity provide an ideal ecosystem for differentiating microorganism communities and microbial biofilms. Biofilm formation respectively includes four main stages (Figure 3): pellicle formation, adhesion, aggregation, and maturation [25]. The structurally and functionally organized biofilm through bacterial succession on any surfaces in the oral cavity—that is not shed—is defined as dental plaque. Including a considerable diversity of microorganism species, the oral microbiota has a key role in protecting the human body by preventing health-affecting extrinsic bacteria from colonization. Losing the balance of this sensitive ecosystem due to immune system failure is proved to be a serious problem facing the systemic health. This imbalance may lead to oral diseases including caries, periodontitis, and gingivitis. The most common strategy for preventing oral diseases is the mechanical removal of biofilms from oral surfaces by regular tooth brushing; however, restorations and dental prostheses are other golden standard [24]. The summaries of therapeutic application of herbal and chemical materials *in vitro* and *in vivo* are presented in Table 1. In the following, the most applied and promising approaches and materials, including biological, chemical, and herbal agents, for preventing oral diseases due to dentine biofilms are reviewed.

## 4. Probiotics

Probiotics are live microorganisms and seem to be the only biological agents used for antibiofilm properties and benefit the host's health at an optimum amount [26]. Although probiotics are mostly well known for gastrointestinal applications, they can also modify the oral environment by competing with cariogenic and pathogenic oral bacteria and interfere with their colonization [27]. Literature implies the regular consumption of probiotics to be substantially effective in preventing or treating dental caries, halitosis, gingivitis, periodontitis, and even oral diseases due to candida infection [26, 27]. Species that can colonize and establish a healthy environment in the oral cavity mainly include *Lactobacillus*, *Bifidobacterium*, and *Streptococcus* species [27]. One mechanism suggested for the antibiofilm function of some commensals in the oral microbiota is producing alkaline compounds that contrast acidogenic bacteria such as *S. mutans* that causes acid stress [28]. The formed biofilms by probiotic bacteria are seen as beneficial because they are considered capable of promoting colonization and long-term stability in the mucosa of the host, preventing contamination by pathogenic bacteria. However, further research in this field is necessary to obtain more reliable evidence.

## 5. Chemical Antibiofilm Materials

### 5.1. Nanoparticles and Nanomaterials

The application of nanoparticles (NPs) as therapeutic agents was a revolution in medicine [29]. Nanomaterials were discovered in the 1980s and, since then, have been used for different purposes in the field of medicine with an extensive perspective of future development [30]. Nanomaterials are used as either antimicrobials for their inherent antimicrobial properties or drug delivery systems specifically designed to have affinity to dental surfaces [31]. Silver (Ag), copper oxide (CuO, Cu_2_O, Cu_2_O_3_, and CuO_2_), zinc oxide (ZnO), titanium oxide (TiO, TiO_2_, and Ti_2_O_3_), graphene (an allotrope of carbon), quaternary ammonium polyethyleneimine (QA-PEI), chitosan (CH), and silica (SiO_2_) nanoparticles are examples of numerous nanomaterials that can control biofilm formation [29, 32–36]. Among all, silver nitrate (AgNO_3_) and silver nanoparticles (AgNPs) are indicated as specific metal nanomaterials with one of the highest capacities to control the oral biofilm [37]. Despite the disadvantage of dentine discoloration by silver nitrate, it is considered a promising approach to coat dentin and prevent biofilm formation on dentin surfaces. AgNP gel can prevent the growth of bacteria and protect teeth from dental plaque formation and secondary caries by disrupting the structural integrity of biofilm created by most oral pathogens such as *E. faecalis* [20, 38]. Silver nanoparticles and silver nitrate can be administered as gel, irritant, and medicament with other materials such as chitosan and calcium hydroxide [28, 38]. Ag-CH-conjugated NPs can reduce biofilm formation contained *Streptococcus* species and *E. faecalis* on implants [24]. On the other hand, mesoporous silica nanoparticles in conjugation with chlorhexidine have a broad spectrum of action [39]. Such NPs have been used with restorative materials for inhibiting biofilm development with no adverse effect on their mechanical properties [40]. An inoculation of fresh *Bacillus subtilis* was used to prepare TiO_2_ nanoparticles. Treatment with 5% TiO_2_-GIC (glass ionomer cement) was most effective in treating dental caries without producing any cytotoxic effects [41]. NaOCl is another antibiofilm material commonly used in endodontic treatment against *E. faecalis* with more irritating capacity compared to the AgNP solution. It is also a good vector for calcium hydroxide (Ca(OH)_2_) to be used in short-term as intracanal medication for removing *E. faecalis* dental biofilms [42]. Biological enzymes are also suggested for their potential of antibacterial function. They perform catalytic functions under strict physiological conditions. However, their broad applications are limited because of some drawbacks. Therefore, synthesis of molecules, complexes, and nanoparticles mimicking natural enzymes has recently been developed as an alternative to natural enzymes. The development of artificial biocatalysts has been accelerated by nanozymes exhibiting the properties of enzymes. Nanozymes offer several advantages over natural enzymes [43]. Synthetic polymers such as polyethylenimine or PEI (also known as polyaziridine) in two linear or branched structural architectures are other biomaterials used for their biocidal effects on oral pathogens. The chemical structure of the linear PEI (LPEI) (containing secondary amino groups) and branched PEI (BPEI) (containing primary, secondary, and tertiary amino groups) accounts for their antibacterial activity (Figure 4) [44]. The eradication of biofilms and resident bacteria using nanoparticles holds great promise. The clinical translation of nanoparticles targeting specific microbial and biofilm features is best done with materials that are nontoxic. The effects of topically applied therapeutic agents on chronic biofilms, such as dental caries, require additional research to characterize.

### 5.2. Modified Dental Materials

Biomaterials have a widespread application in our everyday practice, and they are extensively passed through the next phase of the experiments which is modifications. Research advances indicate that biomaterials precoated with silanes, chlorhexidine, histatins, and antifungal drugs can inhibit biofilm formation at either initiation or development especially on difficult-to-access devices such as dentistry prosthesis [45]. For example, polymeric chlorhexidine-coated implant (the internal chamber) prevents bacterial colonization on the preimplant locations and improve the microbiota quality by reducing species with a higher risk of future restoration failure [7]. Another surface modification is performed by photocatalytic irradiation of TiO_2_-coated biomaterials to kill bacteria on orthodontic wires and implants. Titanium-modified aminopropyl silane is also used for immobilizing active antibiotics such as vancomycin on surfaces [46]. It is vital that new materials are developed to discourage the formation of biofilms. In this study, dental materials that inhibit biofilm formation, inhibit biofilm growth, inhibit microbial metabolism in biofilms, kill biofilm bacteria, and detach biofilms are sought [47].

### 5.3. Arginine

Dietary carbohydrates such as arginine are considered a good supplement with antibacterial effects by limiting their virulence, growth, aggregation, and biofilm formation [48]. Arginine produced by oral commensals is another antibiofilm material used for preventing tooth enamels to be demineralized by oral acidogenic bacteria [28]. Arginine also reduces the biomass of dental polymicrobiota by inhibiting and limiting their colonization [48, 49]. L-arginine specifically prevents *S. mutans* from adherence to the tooth surface by suppressing glucan production and composition resulting in reduced EPS [48, 49]. The arginine function mechanism is creating periods of alkalization that can lead to remineralization and restoring the integrity of the enamel [28]. Oral pathogens such as *Actinomyces naeslundii*, *Actinomyces odontolyticus*, *Aggregatibacter actinomycetemcomitans*, *Enterococcus faecalis*, *Fusobacterium nucleatum*, *Lactobacillus acidophilus*, *Porphyromonas gingivalis*, and *Candida albicans* are shown to be inhibited by protamine which is a polycationic protein rich in arginine residues [48]. The arginine deiminase system (ADS) is a dominant pathway of arginine metabolism that involves oral *streptococci* species (e.g., *S. australis*, *S. cristatus*, *S. gordonii*, *S. intermedius*, *S. sanguinis*, and *S. parasanguinis*), some *Lactobacillus* species, and a few numbers of *Spirochete* species [49]. Recently, an in vitro study indicated that L-arginine (1.5%) could enrich *S. gordonii*, suppress *S. mutans*, and inhibit *P. gingivalis*/*Prevotella oris* coaggregation [48].

Exogenous arginine has been recognized as a promising method for inhibiting biofilm formation, and several arginine-containing products are developed in this regard. An example is arginine-containing toothpaste that has been shown to increase ADS activity in dental caries leading to an oral bacteria composition resembling to that of healthy individuals [49]. 7% arginine added to dental adhesives has been shown to be a safe way to improve the dental biofilm composition without affecting its mechanical properties. Arginine and NaF have offered an ecological control approach on multispecies biofilms since they have shown synergistic preventive effect on *S. mutans*, enriching effect on *S. sanguinis*, and suppressing effect on *P. gingivalis* overgrowth [48]. In a study by Nascimento et al., a HOMIM online analysis tool was used to generate microbial community profiles from the scanned HOMIM arrays (http://bioinformatics.forsyth.org/homim/). A specific taxon in a multispecies sample was detected by a fluorescent spot for that particular probe. The hybridization spots were used to calculate the mean intensity for each taxon. There is a limit of detection of about 104 cells for organisms represented by 0.1% of the total sample. Using this method, Nascimento et al. concluded that toothpaste containing 1.5% arginine can induce dental plaque by increasing arginine availability in the oral environment [50].

### 5.4. Quaternary Ammonium Salts (QAS)

Various composite resin and adhesive systems are common and favorable restorations recognized for their esthetic properties. However, they show about 50% failure rate within ten years mainly due to secondary caries caused by plaque formation. This is while despite the significant improvement mechanical properties and wear resistance of dental composites, their antibacterial properties have remained limited [51]. Then, some efforts such as antibacterial additives (antibiotics, Ag ions, etc.) in the resin and adhesive systems have been made to inhibit secondary caries. QAS are polycations with beneficial traits such as high molecular weight, nonvolatility, chemical stability, low toxicity, and antimicrobial activity against a wide range of microorganisms [52, 53]. Therefore, QAS are firstly used in mouthwash to control oral biofilm in the 1970s; then, they were examined as additives into the resin and adhesive systems and in the 1990s were added into dental composite materials [52, 53]. QAS antibacterial mechanism includes binding to the negatively charged bacterial cell membrane through their positive charge leading to bacterial cell membrane lysis [54].

Recently, the combination of QAS with other compounds has been considered for the development of new composites. Quaternary ammonium dimethacrylate (QADM) is a type of combined QAS with reactive groups on both dimethacrylate ends and can be incorporated into resin without reducing their mechanical features [55]. Also, Imazato et al. have developed a complex QAS (12-methacryloyloxydodecyl-pyridinium bromide or MDPB) with strong antibacterial and antibiofilm effects against *E. faecalis*, *F. nucleatum*, *Prevotella nigrescens*, and *S. mutans* [56]. MDPB has been also used in combination with methacryloxylethyl cetyl dimethyl ammonium chloride (DMAE-CB) and could have limited oral pathogens' growth and adherence [57]. Another copolymer using QAS has been constructed by copolymerizing ionic dimethacrylate (IDMA) and methacrylates such as bisphenol A glycerolate dimethacrylate. The obtained polymers have displayed antibacterial effect on dental composites leading to a reduction of *S. mutans* colonization [58]. Furthermore, IDMA-1 in corporation with silver nanoparticles and calcium phosphate (CaP) particles has been used for developing composite resins and showed augmented bactericidal activity without compromising their mechanical properties [59].

### 5.5. Small Molecules

Interfering the formation of oral biofilm using small molecules with adequate biostability, low effective concentration, and low cytotoxicity is a novel strategy to control dental plaques biofilm formation [59]. The imbalanced homeostasis between the oral microflora diversity and the host's immune system in called dysbiosis. Several products have been studied for treating such microbial imbalance. DMTU (1,3-di-m-tolyl-urea) is a small molecule that can inhibit QS communication system in single or multibacterial species. It has proved inhibitory effects against *S. mutans* biofilm formation as well as multispecies biofilm models. For example, Kalimuthu et al. have used *Streptococcus gordonii* as an early colonizer, *Fusobacterium nucleatum* as a bridge colonizer, and *Porphyromonas gingivalis* and *Aggregatibacter actinomycetemcomitans* as late colonizers to develop a multispecies oral biofilm model and demonstrates the anti-microflora effect of DMTU against the planktonic cells in the multispecies biofilm model [60]. ZY354 is another synthetic small molecule with low toxicity against human oral cell lines and acceptable bactericidal function against common oral *streptococci* (i.e., *S. mutans*, *S. gordonii*, and *S. sanguinis*). A relevant study showed that treating multispecies biofilms with ZY354 reduced demineralizing activity at the interface of biofilm and enamel showing promising potentials for anticaries clinical purposes [61].

## 6. Herbal and Natural Materials in Oral Biofilm Treatments

There are biologically active natural products with uncertain structures that show favorable antibiofilm effects when used as alternative or adjunctive therapies. Polyphenols are examples originated from nature that has at least one aromatic ring with single or several hydroxyl groups and is a group of active compounds found in tea, propolis, cranberry, Galla chinensis, grapes, coffee, and cacao [59]. Chemical, herbal, and natural antibiofilm material mechanisms are described in Figure 5.

### 6.1. Green Tea

Firstly, being popular for its effectiveness in reducing body weight, green tea has medical properties such as anticancer, antioxidant, antiprophylaxis, and antimicrobial as well as anticaries activities. Then, its extract has been used in mouthwash for reducing the bacterial load of saliva (*S. mutans* and *Lactobacilli*) via inhibiting their proliferation, attachment, and some metabolic functions such as acid production of acidogenic species [62]. A main effective component in green tea with antimicrobial properties is catechin whose different types are categorized into four main types: epicatechin (EC), epicatechin-3-gallate (ECG), epigallocatechin (EGC), and epigallocatechin-3-gallate (EGCG). EGC and EGCG constitute the biggest proportions and center most studies showing a variety of antimicrobial properties [63]. Tea catechins also reduce the cariogenic properties of starch-containing nutrients by suppressing the salivary amylase activity [57, 63]. Even in a study by Xue et al., the anticaries and anticariogenicity effects of EGCG have been shown to be associated [57]. Also, the powerful antimicrobial properties of EGCG against *E. faecalis* and *S. mutans* as well as its suppressive effects on their virulence genes have been verified by multiple studies [63].

### 6.2. Propolis

A powerful antifungal and antibacterial agent, propolis also promotes healing of inflammation and has antioxidant properties. A widely studied active component of propolis is caffeine phenethyl ester (CAPE). Antiviral and antibacterial activities are among the many biological activities of CAPE. A previous CAPE study demonstrated effective antifungal action against *C. albicans*. Biofilm formation and hyphal growth of *C. albicans* are inhibited by it as well [64]. Propolis in the form of ethanol extract (EEPs) is an herb-originated nontoxic product that is usually used as a dietary supplement and antibacterial agent [65]. The flavonoids, cinnamic acid-derived material, and bioactive fatty acid contents are considered the main bioactive constituents that inhibit bacterial growth and adherence and exert anticaries effect in propolis [65]. EEP displays an inhibitory effect comparable to chlorhexidine (CHX) against *A. israelii*, *C. albicans*, *Lactobacilli*, *P. gingivalis*, and *P. intermedia* [65, 66].

### 6.3. Garlic

Garlic or *A. sativum* is known as a plant with various antimicrobial compounds. Its extract exhibits inhibitory effects on QS, QS signaling, and virulence factors such as biofilm formation in several microorganisms [67, 68]. N-(Heptylsulfanylacetyl)-L-homoserine lactone is one of the most potent components in garlic that is responsible for interrupting QS signaling and inhibiting QS and some transcriptional regulators (e.g., LuxR and LasR) [69]. The rapid clearing effect of garlic extract in respiratory burst due to tobramycin-sensitive *P. aeruginosa* through phagocytosis by polymorphonuclear leukocytes (PMNs) was found by Bjarnsholt et al. [70]. There are different components of garlic which are presented in Figure 6. Some other phytochemical compounds in the solvent extract of garlic bulb are carbohydrates, proteins, alkaloids, saponins, flavonoids, tannins, and steroids that exert a wide range of antidental caries (Figure 7) [71]. Many studies have approved that the garlic extract has antibacterial, antiviral, and antifungal activities (Figure 8).

### 6.4. Phloretin

Phloretin is a component found in apple with antioxidant, antibiofilm, and antivirulence properties against strains such as *E. coli* O157:H7 and *S. aureus* RN4220 and SA1199B. Phloretin suppresses fimbria production, adhesion to host cells, and the inflammatory response induced by the tumor necrosis factor-alpha, but does not affect bacterial growth in their planktonic phase. Phloretins repress hlyE and stx (toxin genes), lsrACDBFs (autoinducer-2 importer genes), csgA and csgB (curli genes), and prophage genes and also target efflux proteins [72]. According to mentioned study, phloretin may also act as an anti-inflammatory agent in inflammatory diseases and as an inhibitor of biofilm formation.

### 6.5. Limonoids

Limonoids or triterpenoid are secondary metabolites in citrus that interfere with cell to cell signaling, plaque formation, and the type III secretion system in *Vibrio harveyi*, probably via modulating the luxO expression by isolimonic acid and/or ichangin. Isolimonic acid interferes with QseBC/QseA-dependent cell to cell signaling by inhibiting AI-3/epinephrine activation [73]. Biofilm formation can be inhibited by preventing quorum sensing signaling, as can be seen in other compounds later in this article.

### 6.6. Hordenine

Zhou et al. also showed the concentration-dependent decreasing effect of hordenine on signaling molecule production in foodborne pathogen *P. aeruginosa* and block its QS-controlled phenotypes including biofilm formation [73, 74]. The anti-QS function of hordenine is a competitive inhibition toward signaling molecules [74]. Hordenine in combination with nanoparticles (NPs) such as AuNPs has displayed an enhanced antibiofilm effect on *P. aeruginosa* PAO1 [74].

### 6.7. Quercetin

As a plant-originated polyphenol, quercetin shows effective biofilm-limiting, antivirulence, and anticaries properties, namely, against *P. aeruginosa*, *Streptococcus pneumonia*, *S. mutans*, and *E. faecalis* [75]. The quercetin found in fruits, grains, and vegetables suppresses the activity of virulence factors such as pyocyanin and proteases at a much lower effective concentration than that of other herbal extracts and substances [74, 75]. From a mechanismal view, quercetin significantly reduces the expression of QS-associated genes including LasI, LasR, RhlI, and RhlR as well as suppressing sialic acid expression by inhibiting SrtA [75, 76]. These studies explain the potential of quercetin for antimicrobial applications and therapies. Quercetin also shows synergically increased antibiofilm activities in conjugation with nanoparticles that has opened up a novel therapeutic approach for preventing microbial infections [69, 75].

### 6.8. Cranberry

Cranberry is most popular for antibacterial properties owing to its various antioxidant bioactive contents such as anthocyanins, flavonols, flavan-3-ols, phenolic acid derivatives, and tannins [77]. This potential enables cranberry to fight not only cardiovascular diseases and cancer but also a variety of bacterial infections against pathogens including *E. coli*, *Helicobacter pylori*, *Salmonella species*, *S. aureus*, and *S. mutans* [78]. Accordingly, mouthwash products containing the extract of this fruit have reduced the bacteria counts in dental caries and periodontal diseases after daily use [79]. The most active components in cranberry are proanthocyanins (PACs) and flavonols that show a powerful disruptive effect on biofilm formation. The high concentration of purified A-type PAC leads to reducing *S. mutans* biofilm formation and diminishes its acidogenicity [80]. Kim et al. have indicated that PAC oligomers associated with myricetin break down the microarchitecture of cariogenic biofilms, decrease the insoluble EPS amount, and neutralize the acidic microenvironment at the biofilm-apatite interface. These functions cause alternating cell surface molecules, reducing the bacterial hydrophobicity, and prevention of bacterial coaggregation [81]. Polymerization-degree (DP) investigations on PAC oligomer have shown the highest biofilm disruption effect on the bacterial adhesion in DP 4 and DP 8 to 13, especially on smooth surfaces [82–84]. Overall, PACs are suggested as ideal alternatives to or adjunctive for anticaries chemotherapy [85].

### 6.9. Thymoquinone

Black cumin or *Nigella sativa* is an important medicinal plant with treating potentials for a variety of disorders including diabetes, cancer, and reproductive disorders as well as several infectious diseases. Its seeds show anti-inflammatory, antioxidant, immunomodulatory, analgesic, bronchodilatory, hepatoprotective, and spasmolytic properties such as antidiabetic, anticancer, and antimicrobial. Its essential oil components such as thymoquinone (TQ) are responsible for most of its biological activities [86]. In an animal study, Ozdemir et al. fed periodontitis models with thymoquinone and showed a significant reduction in gingival inflammation and alveolar bone loss [86]. These findings warrant further studies on the antibacterial and anti-inflammatory properties of TQ and its potential for preventing periodontal diseases [87]. To explore TQ's use as bioactive substances with antibiofilm potential, further research is needed to examine how it prevents biofilm formation.

### 6.10. *Galla chinensis*

*Galla chinensis* has high content of hydrolyzable tannins and broad bioactive materials including polyphenols (e.g., gallotannin and gallic acid). Both laboratory and animal studies on its extract showed enhanced remineralization of enamel, inhibited growth of caries, and reduced metabolism in pathogens by decreasing the enamel demineralization [88]. Clarification of G. chinensis's exact mechanism and evaluation of its effectiveness have proven difficult. These aspects have been examined in numerous studies: inhibitory effect on oral bacteria, inhibition of demineralization, and enhancement of remineralization, stability, and toxicity [89]. Inhibition of cariogenicity by Galla chinensis is possible. The Galla chinensis plant could be used as a source of new caries-preventive agents.

### 6.11. Other Polyphenol-Containing Plants

There is a wide range of biological activities associated with polyphenols, which are derived from plants. Based on the effects of tea or red wine on glass or cup surfaces, a versatile surface chemistry with polyphenols originated from biomimetic inspiration [90]. Polyphenols are also found in other herbs, namely, cocoa, coffee, hop bract, oat hull, and tea tree or *Melaleuca alternifolia* (MEL). MEL, for example, shows anti-inflammatory and antimicrobial properties against a wide range of microorganisms including bacterial, fungal, and viral species. It has also displayed anticaries and antibiofilm effects against monospecies plaques of periodontopathogens by inhibiting their growth and adhesion. However, its clinical application is limited because of its inadequate clinical stability, water miscibility, and penetrating capacity. Nanotechnology can help remove these limitations and improve its release and selectivity by reducing the size of MEL particles as well as lowering its toxicity [91].

### 6.12. *Mentha piperita*

In Iran and many parts of the world, *Mentha piperita* is a species of the Lamiaceae family that is used for its aroma and therapeutic properties in foods and cosmetic industrial products. Medicinal properties are also found in the leaves and flowers of M. piperita [92]. The antibiofilm potential of *Mentha piperita* essential oil (MPEO) has been studied on *S. mutans*; however, it has shown some other biocidal functions against other bacterial, fungal, viral, and larval species. Interestingly, even high doses (2000 mg/kg) of MPEO have shown no toxicity for humans [82].

### 6.13. *Houttuynia cordata*

*Houttuynia cordata* or Thunberg is a common medicinal herb in Japan. Its poultice has been traditionally used for treating purulent skin diseases, and its ethanol extract has proved antimicrobial and antibiofilm effects on a variety of bacterial species including methicillin-resistant *S. aureus* (MRSA). Regarding the mechanism, stimulation of human keratinocytes occurs by the anti-inflammatory effect of HC that inhibits IL-8 and CCL20 productions. Regarding the potential of HCP in fighting various infections, it is suggested as a therapeutically useful antibiotic and anti-inflammatory modulator for infections or inflammation in the skin with high and long-term effectiveness. Houttuynia cordata poultice ethanol extract was reported to prevent oral infectious diseases, such as periodontal disease, when used as mouthwash for oral care by Sekita et al. [93].

### 6.14. Guava Leaf Extract

*Psidium guajava* or guava tree has extensive medicinal properties. The bioactive components existing in its leaf and bark have valuable therapeutic effects with almost no side effects. The phytochemicals in *P. guajava* leaf include alkaloids, carotenoids, essential and fixed oils, flavonoids, glycosides, lectins, reducing-sugars, saponins, tannins, triterpenes, and vitamins (C&A). Flavonoids and quercetin are the constituents accounting for the antibacterial properties, antioxidant effect and strengthening of the immune system [94]. One mechanism for their anti-inflammatory effect is intervening the production of nitric oxide and prostaglandin E2 induced by lipopolysaccharide [95]. Moreover, the guava leaf extract is suggested to be useful for aphthous ulcers displaying marked pain relief and ulcer resolution effects [94].

### 6.15. *Ligustrum robustum*

*Ligustrum robustum* (Roxb.) Blume is called Ku-Ding-Cha and recognized as a medicinal plant in China where its leaves are used as herbal tea to treat obesity, detoxification, and improving digestion. The Blume's extract has also proved potentials against oxidative stress, inflammation, cancer, infection, and dental caries as well as neuroprotective and hepatoprotective activities with low cytotoxicity. Ligustrum robustum extracts were treated for 24 hours with different concentrations of Ligustrum robustum extracts to test the inhibitory effects on S. mutans UA159 planktonic cells and biofilms by Zhang et al. It was observed in the bacterial growth curve that Ligustrum robustum extracts inhibited bacterial proliferation in a dose-dependent manner, with 0.40% (*w*/*v*) of Ligustrum robustum extracts almost completely inhibiting bacterial growth [96].

## 7. Animal Studies of Chemical Materials in Oral Biofilm Treatments

Dental caries and biofilm formation occur in both animals and humans [97]. Biofilm formation may have several consequences for live organisms that necessitates acquiring more knowledge about their treatments [22]. Accordingly, several studies try to address the anticaries effect of different chemicals on biofilm formation. A turning point in this regard was a dual strategy using microarc oxidation + poly (amidoamine)-loading dimethylaminododecyl methacrylate (PD) to combat biofilm formation that achieved promising results against peri-implantitis [87, 98]. Prates et al. stated that using protoporphyrin derivative as an antimicrobial photodynamic therapy agent exhibits 30% dental bone recovery [99]. Moreover, poly (ethylene) glycol-poly (*β*-amino esters) micelles have been conjugated with other antimicrobials and could fairly eradicate *S. aureus* infection [100]. The impact of antibiotics and NO-releasing biomimetic nanomatrix gel on different bacterial biofilms has been assessed by Choi et al. and indicated a concentration-dependent antibacterial effect [101]. Despite variations in chemical structures and collection from different geographical regions, Kharshid et al. clearly established that propolis exhibits remarkable antibacterial properties. This natural resin shows limited activity against gram-negative bacteria, although it seems to be effective against gram-positive rods and *M. tuberculosis*. It was shown that propolis extract is cariostatic in at least three different aspects of caries development, *S. mutans* vulnerabilities, and the activity of glycosyltransferase in rats, in three different studies [66]. Finally, the results of the evaluation of dental hygiene chew and 0.2% *W*/*V* chlorhexidine on dental plaque formation in dogs have been successful [102]. Although there are few exceptions where the intervention has not achieved its primary endpoint, the results are generally promising.

## 8. Clinical Studies of Chemical Materials in Oral Biofilm Treatments

As the archetypical biofilms, dental plaques are composed of a heterogeneous community of microbes that underlies many dental and periodontal diseases including dental caries. The balance between the periodontal pathogens and the host immune system determines the clinical representation of dental diseases. If the delicate balance and harmonious relationship of plaque and adjacent tissues are disturbed, the healthy state between them will be ruined and the disease will appear [103]. Patients' oral hygiene home care performance can be measured and motivated using disclosing agents. “Colorimetric technique” describes this method. It is important to apply the disclosing agent correctly and with the right technique. The clinician can motivate patients to prevent periodontal disease by using disclosing agents to reveal the areas around the teeth, including bacterial biofilm [104]. Evaluation of the clinical facet of dental biofilm formation is mentioned in several studies. For example, sucrose exposure to the biochemical and microbiological composition of dental biofilm showed its positive effect on enamel demineralization especially in the presence of fluoride [105]. Moreover, controlling the dental biofilm can be improved by adding a vegetable or mineral oil to dentifrice that confirms the associated benefits of treatments containing essential oils [106]. Similarly, a combination of chlorhexidine, fluorine, and erythrosine has decreased the dental biofilm and gingival bleeding in patients with Down syndrome [107]. Triclosan toothpaste has been evaluated for modulation of the clinical and subgingival condition in children from aggressive periodontitis parents and could effectively control the periodontal parameters and enhance the immune factors in subjects [108]. In another study, a temporal relationship was shown between biofilm composition and enamel demineralization following exposure to sucrose. The findings indicated that sucrose affects the insoluble extracellular polysaccharides differentially higher than monosaccharide components, and changes in the biofilm composition occur earlier than enamel demineralization [109]. Finally, these results verified the clinical implications of chemical treatments for dental biofilms (Table 2).

## 9. Clinical Studies of Herbal Materials in Oral Biofilm Treatments

Considering the important role of dental biofilm in oral health and the approved positive effect of herbal materials, several studies have evaluated the effect of medicinal herbs on dental biofilm. Clinically, a mouth rinse containing guava leaf extract was shown to be a useful adjunct to professional oral prophylaxis for chronic generalized gingivitis [94]. In another study, the inhibitory effects of chlorohexidine and MEL nanoparticles against biofilm and inflammation showed similar results on tooth surfaces free of or covered by biofilm [91]. Another randomized clinical trial study used an experimental solution of *Ricinus communis* through a cleansing regimen on a silicone-based denture liner to assess the integrity of liners and showed antibiofilm and antimicrobial effects of solution [110]. Saliasi et al. compared the potential of two dentifrice in reducing the interdental gingival bleeding. One of their used mouthwash contained *Carica papaya* leaf extract (CPLE) and the other one was a classical sodium lauryl sulfate- (SLS-) free dentifrice containing enzyme. This study indicated that CPLE more efficiently reduced the gingival bleeding and inflammation compared to the classical SLS-free dentifrice [111]. In another study, four antimicrobial mouth rinses in different formulations were tested for their effects on the clinical parameters of adjacent tissues and subgingival microbiota composition. The alteration in the composition of subgingival microbiota made by the studied mouth rinses improved the clinical parameters [112]. Collectively, the above-mentioned findings confirm that herbal medicines can be considered important effective agents in treating dental biofilms (Table 2).

## 10. Clinical Studies of the Mixed Materials (Herbal and Chemical) in Oral Biofilm Treatment

Nearly 1000 species of bacteria live in the mouth. In treating caries, hard tissues are usually restored in regard to functional and aesthetic concerns. Nonetheless, this treats only the outcomes of the illness. Typically, in clinical settings, contaminated tissues are removed to prevent the spread of dental caries [113]. Dental materials are designed to kill microbes in contact by strategically incorporating a wide range of antimicrobial agents (such as polycations, quaternary ammonium compounds, and antimicrobial peptides). Covalent compound structures can be formed by combining the compounds with dental materials. Both gram-negative and gram-positive bacteria are strongly affected by these broad-spectrum antimicrobial agents [4]. Recently, antimicrobial dental materials have been prepared using QAMs and AgNPs. In addition to killing bacteria on the surface, the modified materials also kill bacteria away from the surface [3]. An evaluation of barley hordenine, a polyphenolic compound, as well as a combination with netilmicin, an aminoglycoside antibiotic, was carried out by Zou et al. (2018). In a study using hordenine and netilmicin together, up to 88% of *P. aeruginosa* PAO1 biofilms were reduced, compared to none of the treatments individually [74]. In order to target biofilms more effectively, studies should combine natural antibiofilm compounds from different sources. Moreover, natural compounds are not effective against all bacterial strains, so selecting an effective compound is also necessary [114].

## 11. Conclusion

Supported with strong clinical efficacy proof, antibiofilm materials are being increasingly considered and applied as efficient agents for controlling the dental biofilm and ameliorating gingivitis. However, generally, herbal-based materials produce a lower score in comparison to mouthwashes containing chemical materials such as CHX, fluoride, and EO. In addition, the importance of mechanical removal is still on the top priority among all dental biofilms controlling methods and chemical treatment provides an alternative or adjunctive method by preventing biofilm accumulation rather than oral microflora eradication. The present study reviewed that factors beneficial in preventing dental caries include probiotics, herbs, and spices. Also, it indicated that combining multiple plants or plants with probiotics can exert more efficient results than individual therapies using single herbal products or probiotics. Surveying the literature showed that probiotics act not only as possible antimicrobial agents but also sustain the oral ecosystem's balance. Finally, the combination of functional products containing probiotics and polyphenol extracts is an important research trend in the food industry.

## 12. Future Direction

This review highlighted the recent successful studies on using antibiofilm chemical and herbal materials. Nevertheless, several problems and limitations remained to be addressed. The majority of evidence results from laboratory or preclinical trial studies in short-time projects, whereas longer-time studies are required to provide more reliable quantitative proof that confirms techniques have benefits in vivo and verify that their antibacterial effect is durable. On the other hand, the safety profile of the above-mentioned antimicrobial agents and the emergence of antimicrobial tolerance as a major concern require further investigation. In addition, well-planned and appropriately structured clinical trials conducted across multiple centers are required for accurate comparisons. Such extensive trials are also essential to find the most efficient antimicrobial or antibiofilm approach and suitable criteria for opting them in. Furthermore, the potential synergic functions of nature-originated materials and chemical agents should be targeted in future studies. Such studies and information are necessary to develop novel, efficient, and healthy anticaries strategies. In the end, the biofilm-interfering or biofilm-inhibiting activities of these products should be investigated in cohort clinical trials. Several herbal materials as well as their active ingredients need further study and clarification with regard to their antimicrobial and antioxidant properties.

## Figures and Tables

**Figure 1:** QS mechanism in gram-categorized species. The canonical QS signaling and the Agr system are the most typical processes involved in the biofilm formation in gram+ bacteria *S. aureus*. This system includes four genes (AgrA-D) under the control of one operon. The products of this operon include virulence factors such as toxins and proteases. AgrD is converted to autoinducer peptides (AIPs) during secretion through AgrB to out of the cell where it activates the transmembrane AgrC by phosphorylation. The activated AgrC further activates AgrA that promotes the expression of targeted genes by influencing two promoters (P2 and P3). P2 regulates the Agr operon system, and P3 activates the expression of RNAIII which is the key regulator of different factors relating QS and biofilm formation. RNAIII upregulates virulence factors and inhibits factors contributing to bacterial dispersal. The balancing function Agr proteins on bacterial swarming and infection makes them promising targets for developing therapeutic antibiofilm agents [69].

**Figure 2:** QS mechanism in gram-categorized species. In gram− bacteria biofilm formation, QS signaling involve autoinducer acyl-homoserine lactones (AHLs) that help communication among bacteria and modulate targeted genes expression by activating corresponding cytoplasmic receptors. The Luxl/luxR transcriptional factors are other essential regulating factors activated by AHLs and control the expression of various virulence factors in different gram− bacteria such as pigments, carbohydrate-binding proteins, various proteases such as elastase, toxin, different autoinducers such as *Pseudomonas* quinolone signal (PQS), CAI-1, and AI-2, as well as QS receptors such as LasI/LasR, RhlI/RhlR, CqsS, and LuxPQ. Specific autoinducers can also further promote other adhesives and virulence factors [69].

**Figure 3:** The four main stages of biofilm formation process in the oral cavity [25].

**Figure 4:** The synthesis of (a) linear polyethyleneimine and (b) branched polyethyleneimine [44].

**Figure 5:** Antibiofilm activities and mechanisms of herbal and neutral materials.

**Figure 6:** Different components of garlic [71].

**Figure 7:** Structure of important bioactive constituents present in garlic [71].

**Figure 8:** Antibacterial, antiviral, and antifungal activities of extract of garlic.

**Table 1:** *In vivo* and *in vitro* studies in oral biofilm treatments.

Type	Method	Outcomes	Year/Ref
Herbal materials			
Apple-boysenberry beverage	Quantitation of Lactobacillus spp., *A. naeslundii*, and *S. mutans* in saliva samples using qPCR	The bioactive beverage reduced the proliferation of *Actinomyces* and *Streptococci* down to almost half.	2017/ [115]
Cranberry proanthocyanidins	The antibiofilm and anticaries effects of proanthocyanidin's against *S. mutans* was assessed in vitro and in vivo, respectively.	Proanthocyanidin treatment inhibited smooth-surface caries in rats.	2010/ [80]
Toothpaste and mouth rinse containing natural/herbal agents	Six commercially available products were compared to PBS as control on artificial plaque in animal model.	Four mouth rinses (Tom's Propolis & Myrrh®, Colgate Total 12® toothpaste, Malvatricin® Plus, and PerioGard®) significantly reduced the biofilm viability.	2019/ [116]
*Zingiber officinale*	The crude and methanolic extracts of ginger were evaluated at sub-MIC levels on *S. mutans* caries in vitro and in vivo.	Both extracts showed strong anticariogenic effect.	2015/ [117]
*Roselle calyx*	The antibacterial activity of the herbal extract was studied on eight oral bacterial strains in vitro.	The extract showed antibacterial activity especially against *F. nucleatum*, *P. intermedia*, and *P. gingivalis*.	2016/ [118]
*Terebinthifolius* and *Croton urucurana*	The antiadherent and antibiofilm potentials of plants were studied in vitro by evaluating their minimal concentration of adherence (MICA).	Both herbal extracts inhibited *S. mutans* and *C. albicans from forming* biofilm.	2014/ [119]
Garlic	The MIC of garlic extract against *S. mutans* was studied in vitro.	Garlic extract increased the biofilm formation of *S. mutans* on the orthodontic wires.	2011/ [120]
Limonoids	The antibiofilm activity of limonoids against *Vibrio harveyi* was evaluated in vitro.	Limonoids showed significant modulatory functions interfering with biofilm formation.	2011/ [73]
Hordenine	The inhibitory activity of hordenine against quorum sensing was studied using high-resolution microscopy and RT-PCR.	Hordenine inhibited quorum sensing of foodborne pathogens by competing with their signaling molecules.	2018/ [74]
Quercetin	The effect of quercetin on *P. aeruginosa* biofilm and virulence factors was studied in vitro.	Quercetin effectively inhibited the biofilm formation and reduced *P. aeruginosa* virulence.	2016/ [75]
Red wine Dealcoholized red wine Red wine extract (with or without grape seed)	The effect of seed extract on an oral supragingival plaque model was studied in vitro and using high-resolution microscopy.	Solutions spiked with seed extract showed antimicrobial effect on 3 of 5 studied strains (*F. nucleatum*, *S. oralis*, and *A. oris*). Red wine and dealcoholized wine showed antimicrobial effects on 2 strains (*F. nucleatum* and *S. oralis*).	2014/ [121]
*Myristica fragrans*	MIC and MBC tests were performed using the ethanol and ethyl acetate extracts of seed and mace of plant in vitro.	The ethanol extract of the plant displayed better antimicrobial potential compared to the ethyl acetate extracts.	2012/ [122]
*Olea europaea*, *Inula viscosa*, and mastic gum	MIC and the MBC assays were performed against oral microbiota (10 bacteria and 1 yeast) in vitro.	The most considerable antimicrobial effect belonged to the ethyl acetate extract of *I. viscosa* and the total extract of mastic gum.	2014/ [123]
The essential oils of *Citrus limonum* and *Citrus aurantium*	The antibiofilm effect was studied in vitro against *C. albicans*, *E. faecalis*, and *E. coli*.	Both essential oils displayed antibiofilm effects against all species.	2014/ [124]
The commercially available essential oils of 15 plants	MIC and MBC test against a panel of oral bacteria was performed in vitro.	The essential oil of *Cinnamomum zeylanicum* displayed a moderate antimicrobial effect on *Fusobacterium nucleatum*, *Actinomyces naeslundii*, *Prevotella nigrescens*, and *Streptococcus mutans.*	2016/ [125]
Aqua extract of *Hypericum perforatum*	Colorimetry, microtitration, and resazurin assays were performed using *S. mutans*, *S. sobrinus*, *L. plantarum*, and *E. faecalis.*	The extract showed high antibacterial potential against *S. sobrinus* and *L. plantarum* but moderate antibacterial potential against *S. mutans* and *E. faecalis*.	2016/ [126]
Essential oils extracted from 8 Guatemalan medicinal plants	MIC assay was exerted in vitro on *S. aureus*, *E. coli*, *S. mutans*, *L. acidophilus*, and *C. albicans*.	*S. mutans* showed high sensitivity to all used essential oils. *C. albicans* was sensitive to 4 species.	2015/ [127]
*Ligustrum robustum*	In vitro microbial tests and high-resolution microscopy were used to assess the effect of herbal extract against *S. mutans* biofilm and exopolysaccharide formation.	The extract downregulated the expression of quorum sensing factors and genes encoding glucosyltransferase in *S. mutans*.	2021/ [96]
Quercetin Kaempferol	MIC and MBC assays were evaluated in vitro using *S. mutans*.	These materials reduced biofilm formation, protein expression, cell proliferation, and glucan production.	2019/ [128]
*Houttuynia cordata* ethanol extract (wHCP)	The antimicrobial and antibiofilm potentials of a water solution of extract were evaluated on a number of oral pathogens in vitro.	wHCP showed limited antimicrobial potential but high antibiofilm effects against *F. nucleatum*, *S. mutans*, and *C. albicans*.	2016/ [93]
*LongZhang gargle*	The antibiofilm and antiacid effects of *LongZhang gargle* on *S. mutans* were evaluated in vitro.	*LongZhang Gargle* displayed a significant antimicrobial activity.	2016/ [129]
*Equisetum giganteum* *Punica granatum*	In vitro microbial tests and microscopy were used to test herb extracts' potential against *Candida albicans*.	Herb extracts synergized the antibiofilm effect of adhesive materials.	2018/ [130]
*Azadirachta indica* *Mimusops elengi* *Chlorhexidine gluconate*	The remaining microbial load on the extracted tooth sections after the antimicrobial treatment was evaluated in vitro.	Herb extracts displayed significant antimicrobial effects.	2015/ [131]
*Mangifera indica* *Ocimum sanctum*	*E. faecalis* planktonic growth was tested in vitro.	Herb extracts significantly reduced the growth amount.	2013/ [132]
*Mentha piperita* essential oils	The molecular effect of sub-MIC volume of the essential oil loaded on a chitosan nanogel was evaluated on biofilm formation-associated gene expression of *S. mutans*.	The expression levels of gtfB, gtfC, gtfD, gbpB, spaP, brpA, relA, and vicR genes showed alterations.	2019/ [82]
Methanolic extracts of *Myrtus communis L.* and *Eucalyptus galbie*	The antibiofilm effects of MIC and MBC levels of herb extracts were evaluated on *Enterococcus faecalis*.	The herb extracts had significant antimicrobial potential.	2019/ [133]
*Piper nigrum* *Piper longum* *Zingiber officinale*	Molecular tests were used to assess the antibacterial effect of herbal and chemical medicaments against *E. faecalis*.	The herb extracts showed antibacterial activity lower than calcium hydroxide and higher than saline.	2019/ [134]
*Galla chinensis extract* (*GCE*)	The extract was applied to the polymicrobial plaque model in vitro.	GCE inhibited excess acid production by the biofilms.	2012/ [88]
*Nigella sativa Lin.*	The effect of herb oil was studied on *Fusobacterium nucleatum* and *Actinomyces naeslundii* biofilm formation in vitro and using high-resolution microscopy.	Thymol and thymoquinone (the active constituents of herbal oil) have an inhibitory effect on biofilm formation.	2020/ [87]
*Garlic extract*	Three concentrations of herb extract were examined on *E. faecalis* biofilm formation.	The biofilm production significantly decreased in a concentration-dependent manner.	2015/ [135]
*Triphala*	The antibiofilm effect of herb extract against *S. mutans* was studied ex vivo on tooth substrate.	*Triphala* significantly reduced the biofilm formation by *S. mutans*.	2014/ [136]
Chemical materials			
Ethanolic extract of Polish propolis (EEPP)	Clinical-isolated coagulase-negative *staphylococci* and *S. epidermidis* were used for assessing the antibacterial activity of EEPP in vitro.	EEPP reduced bacterial growth and biofilm formation.	2013/ [137]
Chlorhexidine varnish	Digital photography was used in orthodontic patients.	Chlorhexidine varnish decreased bacterial growth.	2015/ [138]
Erythritol powder	Periodontal therapy was performed for six months, and microbial/clinical outcomes were assessed in the clinic.	Compared to GPAP, EPAP was less abrasive and produced smaller particles.	2015/ [139]
Dentifrice containing *Eugenia uniflora*	The antibacterial effect of the dentifrice on 3 oral bacteria (*S. mutans*, *S. oralis*, and *L. casei*) was examined in vitro.	The tested dentifrice had significant antibacterial effect.	2016/ [140]
Methylene blue-loaded poly(lactic-co-glycolic) nanoparticles (MB-NP)	MB-NP was applied to multistrain dental biofilm in vitro and followed by photodynamic therapy (PDT).	The combination of MB-NP and PDT resulted in improving clinical parameters.	2016/ [141]
MB-NP	Dental plaques underwent PDT in a clinical pilot study. Planktonic and biofilm phases were assessed in vitro.	PDT was confirmed as a safe treatment that improved clinical parameters.	2016/ [141]
Stannous fluoride and zinc citrate dentifrice	Mineralized biofilms were used to examine the antibiofilm potential of mouthwash in vitro and in vivo.	The used dentifrice decreased calcium accumulation in the biofilm.	2017/ [142]
Stannous fluoride or triclosan dentifrices	The effects of two dentifrices on oral biofilm models (acid production/glycolysis inhibition) and plaque growth were assessed in vitro and in vivo, respectively.	Stannous fluoride dentifrice significantly reduced glycolysis and plaque growth.	2017/ [143]
3 commercially available kinds of toothpaste Chlorhexidine	The bactericidal effect of materials on a baseline biofilm flora was examined in vitro.	All kinds of toothpaste showed significant bactericidal effects but were lower than the chlorhexidine mouth rinse.	2018/ [144]
Doxycycline hyclate-containing resin	*S. mutans* microbial load was evaluated after a 3-month clinical trial.	The composite resin could eliminate all bacteria.	2018/ [145]
Toothpaste containing zinc oxide, zinc citrate, and L-arginine	All silica-based kinds of toothpaste were used on the oral bacteria on the teeth, tongue, cheeks, and gums.	The designed product could significantly reduce bacterial load in all samples.	2018/ [146]
Polysiloxane- and chlorhexidine-containing alcoholic solution	The bacterial load on bilateral fixed prostheses or crown restorations with a medicament-coated internal chamber was tested in a clinical study by molecular assays.	Polymeric chlorhexidine-coated implants displayed a limiting effect on the bacterial load of the peri-implant tissue.	2019/ [7]
Propolis solution Alkaline peroxide	Digital photography and microbiological quantifications were performed on *Candida spp.* and *S. mutans* biofilms.	Both materials displayed significant bactericidal and antifungal effects.	2019/ [147]

**Table 2:** Clinical studies in oral biofilm treatments.

Type	Method	Outcomes	Year/Ref
Herbal materials			
Allium tuberosum Coriandrum sativum Cymbopogon martini Cymbopogon winterianus Santolina chamaecyparissus	MIC of extracts and essential oils and their antibiofilm effect against *C. albicans* were evaluated in vitro. Chromatography, spectrometry, and scanning electron microscopy (SEM) were used for biochemical evaluations.	The *C. sativum* essential oil and crude oil inhibited biofilm formation and growth.	2011/ [148]
*Aloe vera* gel	The antimicrobial effect of *Aloe vera* gel against some oral pathogenic bacteria was evaluated in vitro.	An optimum concentration of *Aloe vera* gel displayed significant antiseptic function against dental and periodontal pathogens.	2012/ [149]
*Equisetum arvense L.* *Glycyrrhiza glabra L.* *Punica granatum L.* *Stryphnodendron barbatimam*	The antibacterial effect and cytotoxicity of plant extracts were tested in vitro.	All plant extracts displayed antibacterial effect. *E. arvense L. extract* and *G. glabra L. extract* showed the highest and lowest cytotoxic effect, respectively.	2013/ [150]
Mouth rinse containing *Acacia nilotica*	The antibacterial effect of *Acacia nilotica* was evaluated against *S. mutans* in a clinical trial recruiting volunteer.	*A. nilotica* significantly decreased the bacterial load.	2015/ [151]
Green tea *Salvadora persica L.* aqueous	Antibacterial effect of the combined mouthwash was evaluated against plaque accumulation.	The combined mouthwash significantly decreased plaque formation.	2016/ [152]
Phloretin	The effect of flavonoids on the growth and biofilm formation of *S. aureus* strains was evaluated in vitro.	Even sub-MIC values of flavonoids could inhibit the biofilm formation.	2017/ [72]
*Ricinus communis* and sodium hypochlorite	The antimicrobial effect was evaluated using molecular methods.	The denture cleanser effectively inhibited biofilm formation by *C. albicans*.	2017/ [153]
Propolis Chlorhexidine	Antioxidative and antibacterial effects of both materials were compared by evaluating clinical parameters.	Propolis-based formula showed similar clinical chlorhexidine.	2018/ [154]
*Carica papaya* leaf extract	Clinical outcomes were evaluated during a 4-week treatment period.	The herb-containing dentifrice showed similar effect to other used mouthwashes on the gingival bleeding.	2018/ [111]
*Juglans regia L.*	Antibacterial effect of herb extract against *P. aeruginosa* isolated from burn, tracheal, and urine infections was evaluated in vitro.	The herb extract displayed antibiofilm effect on a concentration-dependent manner.	2018/ [155]
*Melaleuca alternifolia* nanoparticles mouthwash with chlorhexidine gluconate	Plaque and gingival clinical parameters as well as participants' perceptions were assessed in recruited subjects.	Chlorhexidine resulted in a better taste, higher antibiofilm effect, and more taste change.	2019/ [91]
Mouth rinse containing *guava* leaf extract	*Guava* was compared to chlorhexidine in terms of antimicrobial and antioxidant effects by clinical and microbial assessments.	*Guava* leaf extract showed similar antibiofilm effects compared to chlorhexidine.	2019/ [94]
*Melaleuca alternifolia*	The effect of herb was compared to chlorhexidine in terms of clinical parameters.	The anti-inflammatory potential of two materials displayed to be similar.	2019/ [91]
Probiotic yogurt containing *Bifidobacterium lactis* Bb12	Antibacterial effect of probiotic yogurt on salivary bacteria was evaluated.	The probiotic yogurt significantly reduced the salivary bacteria.	2020/ [156]
*Ricinus communis* Chloramine-T Sodium hypochlorite	The antimicrobial effect against *Candida spp.* was compared among the three material counts by clinical assessments and photography.	All materials improved denture stomatitis and reduce biofilm formation while sodium hypochlorite had the highest efficacy.	2020/ [157]
Leaf extracts of *Citrus hystrix DC*, *Moringa oleifera Lam*., and *Azadirachta indica A. Juss.*	The effect of herb extracts was studied on gingivitis and compared to chlorhexidine gluconate in terms of clinical and oral microbial parameters.	*Moringa oleifera Lam.* significantly reduced gingivitis and plague. *Azadirachta indica A. Juss.* showed high antimicrobial effect against *Staphylococcus* and *Candida* strains.	2021/ [158]
Chemical materials			
Mouthwash containing essential oils	Biofilms were stained and analyzed by microscopy.	Bacterial vitality was reduced significantly.	2015/ [159]
Taurolidine Chlorhexidine	The efficacy of treatments on biofilm removal was evaluated using clinical outcome parameters.	Taurolidine enhanced antibiofilm effect.	2015/ [160]
Glycine powder Sodium bicarbonate	Both materials were used as air polishing. Gingival and clinical parameters were evaluated.	Glycine powder air polishing significantly improved the measured parameters.	2015/ [161]
Polymethyl-methacrylate and Ag nanoparticles	Antibacterial potential of two formulations against cariogenic bacteria was assessed.	Both formulations inhibited biofilm formation of all tested bacteria.	2015/ [162]
Toothpaste containing fluoride and fluoride plus sodium trimetaphosphate	The antibiofilm effect of toothpaste was assessed.	The formulations containing sodium trimetaphosphate showed higher antibiofilm potentials.	2015/ [163]
Triclosan formula	The antiplaque effects were assessed in vitro.	Including triclosan in formulation significantly inhibited plaque formation.	2015/ [164]
Floss impregnated with chlorhexidine gluconate	Antibiofilm effect was assessed on 4 different surfaces (mesiobuccal, distobuccal, mesiolingual, and distolingual).	Chlorhexidine-impregnated floss displayed synergic reducing effect on supragingival biofilm.	2015/ [165]
Chlorhexidine gluconate Essential oils Cetylpyridinium chloride Triclosan *Hamamelis virginiana*	The inhibitory effect of all materials against bacterial plaque was evaluated.	All mouthwashes containing the five ingredients significantly reduced the biofilm formation.	2015/ [166]
Mouthwash containing *Matricaria chamomilla L.* and chlorhexidine	Clinical parameters were evaluated in a clinical trial.	The mouthwash significantly reduced the visible plaque formation and gingival bleeding.	2016/ [167]
Triclosan	Clinical parameters were evaluated in a clinical trial.	No considerable change occurred in the plaque and gingival indexes of triclosan-treated subjects.	2016/ [168]
Sodium perborate Chlorhexidine	The antibiofilm effect of disinfection agents was assessed in vitro.	Brushing combined with agents successfully inhibited biofilm formation on dentures.	2016/ [169]
Stannous fluoride (SnF_2_)	Dental plaque was sampled and evaluated in terms of gingival inflammation and bleeding.	SnF_2_-containing dentifrice improved clinical outcomes of gingivitis and plaque.	2017/ [170]
—	Scaling and root planing with or without laser diode was assessed in terms of clinical, microbiological, and inflammatory effects.	Diode laser synergically improved parameters.	2017/ [171]
Chlorhexidine solutions	The antiplaque effect on clinical samples was examined in vitro.	The treatment significantly prevented plaque and subgingival biofilm formation.	2017/ [172]
Acidulated phosphate fluoride	The antibiofilm effect against salivary *S. mutans* was studied in vitro after topical application.	The treatment displayed no inhibitory effect on salivary or biofilm bacterial load.	2017/ [173]
Toothpaste containing arginine	Some biochemical and microbial parameters were evaluated.	The treatment reduced lactic acid production.	2017/ [174]
Fluoride-impregnated toothbrush Fluoride-containing toothpaste	The remained fluoride in saliva and antiplaque effects were evaluated on buccal and lingual surfaces.	Both treatments displayed similar plaque-removing outcomes.	2017/ [175]
Saline Sodium hypochlorite Ricinus communis	The antibiofilm effect against *Candida spp.* on the intaglio surface of maxillary dentures was evaluated using photography and quantifying software.	Only different concentrations of sodium hypochlorite displayed antimicrobial effect.	2017/ [176]
Hyaluronic acid mouthwash Chlorhexidine	Plaque and clinical parameters were evaluated in clinics.	The mouthwash showed a marginally less inhibitory effect on plaque formation compared to chlorhexidine.	2017/ [176]
Silver/fluoride nanoparticles	The bactericidal and antibiofilm effects were evaluated on *S. mutans*.	Nanoparticles were reported to be effective and suggested for clinical application in order to limit dental biofilm formation.	2017/ [177]
Mouth rinse containing chlorhexidine gluconate	Antimicrobial effect against *S. mutans* was analyzed using microscopy.	The intense contamination showed no significant difference in the microbial load.	2017/ [178]
Probiotic (*B. lactis*)-containing lozenges	Lozenges were used with scaling and root planning. Clinical, immunological, and microbial parameters were monitored.	The treated subjects displayed higher antibacterial and lower inflammatory effects.	2018/ [179]
Propolis/herbs in antioxidant-based formula Chlorhexidine-based formulae	A couple clinical parameters were monitored in a 3-month trial study.	The two formulas displayed similar clinical outcomes.	2018/ [154]
Sodium bicarbonate	A couple clinical parameters were monitored in a clinical trial.	Sodium bicarbonate displayed increasing antibacterial effect.	2018/ [180]
Modified antimicrobial peptide	A couple clinical parameters were evaluated in a clinical trial.	The modified peptide displayed antibacterial effect against periodontal bacteria.	2018/ [180]
Fluoridated dentifrice containing arginine	A couple clinical and microbial parameters were examined.	Arginine did not display any additional antibiofilm effect.	2018/ [181]
Edathamil-containing gel	Antiplaque effect was evaluated by photography.	Edathamil increased the plaque removal.	2018/ [182]
Toothpastes containing different concentrations of sodium bicarbonate	Antiplaque effect was measured before and after a single-timed brushing.	No statistically significant difference was observed.	2018/ [183]
Dentifrices containing different ratios of sodium fluoride and tara gum	The fluoride concentration was determined using a physicochemical technique.	The antibiofilm effect displayed no statistically significant differences.	2018/ [184]
Chlorhexidine digluconate-impregnated dental floss	The plaque index was assessed in clinics.	The impregnated floss significantly reduced the plaque formation.	2018/ [185]
Metronidazole Amoxicillin	Subjects were treated with systemic antibiotic as an adjuvant therapy, and antibiofilm outcome was evaluated.	No significant differences were observed in clinical parameters.	2019/ [186]
Arginine- or fluoride-containing toothpastes	Caries diagnosis and plaque sampling were performed on tooth surfaces, and antiplaque effects were evaluated in vitro.	The arginine deiminase system was significantly activated, and the acidity was reduced in the plaque. Fluoride reduced plaque lactate production.	2019/ [187]
Sodium hypochlorite Chlorhexidine gluconate Sodium bicarbonate	Antimicrobial activity was quantified in healthy complete denture wearers through chemical analysis.	Sodium hypochlorite and chlorhexidine significantly decreased microbial viability.	2019/ [188]
Lozenges containing probiotic *Streptococcus salivarius* M18	Plaque and gingival outcomes were measured in orthodontic brace wearers using molecular analyses.	Treatment had no effect on microbial parameters.	2019/ [189]
Mouth rinses containing chlorhexidine and guava	Plaque and gingival indexes were measured.	Plaque and gingival indexes as well as microbial counts showed gradual reduction.	2019/ [94]
Triclosan toothpaste	Plaque and gingival indexes were measured.	Triclosan toothpaste displayed antiplaque effect.	2020/ [108]
Triclosan toothpaste	Plaque index and gingival bleeding were measured.	Treatment with triclosan toothpaste reduced gingival bleeding and plaque formation.	2020/ [190]
Sodium hypochlorite gel	Pocket probing depth was evaluated before and after treatment.	No statistically significant difference was observed.	2020/ [191]
Sodium hypochlorite Dettol and Lifebuoy liquid soap Phosphate-buffered saline	The antimicrobial effect against *Candida spp.* was evaluated in vitro.	All three treatments significantly reduced the microbial load.	2020/ [192]
Ozonated water	The antiplaque and antibiofilm effects were assessed in vitro.	No statistical difference was observed.	2021/ [193]
Mouth rinses containing chlorhexidine with or without hydrogen peroxide	The antiplaque effect was studied in vitro.	Both mouth rinses significantly controlled the plaque formation. Hydrogen peroxide had a slightly synergistic effect.	2021/ [194]

## Data Availability

This article is a review and does not contain any studies with humans or animals performed by any of the authors.
